This article has been retracted.

# Molecular Characterization and Antibiotic Susceptibility Pattern of Bacterial Strains Isolated From Wound of Patients With Diabetes

**DOI:** 10.7759/cureus.47681

**Published:** 2023-10-25

**Authors:** Eemaz Nathaniel, Jibran Ikram, Aimen James, Bakhtawar Obaid, Ayesha Zahid, Zeeshan Ahmed, Dilawar K Wazir, Qazi Muhammad Farooq Wahab, Giustino Varrassi, Satesh Kumar, Mahima Khatri

**Affiliations:** 1 Research, Rehman Medical Institute, Peshawar, PAK; 2 Orthopaedics and Trauma, Rehman Medical Institute, Peshawar, PAK; 3 Dermatology, Rehman Medical Institute, Peshawar, PAK; 4 Internal Medicine, Rehman Medical Institute, Peshawar, PAK; 5 Surgery, Rehman Medical Institute, Peshawar, PAK; 6 Medicine, Hayatabad Medical Complex Peshawar, Peshawar, PAK; 7 Microbiology, University of Peshawar, Peshawar, PAK; 8 Medicine, Khyber Teaching Hospital, Peshawar, PAK; 9 Pain Medicine, Paolo Procacci Foundation, Rome, ITA; 10 Medicine and Surgery, Shaheed Mohtarma Benazir Bhutto Medical College, Karachi, PAK; 11 Medicine and Surgery, Dow University of Health Sciences, Karachi, PAK

**Keywords:** cross-sectional study, wound infections, antibiotic susceptibility, molecular characterization, bacterial strains, diabetic patients

## Abstract

Background: Diabetic wound infections are susceptible to various pathogens, particularly bacteria, due to the immunocompromised state of diabetic patients. *Staphylococcus aureus* is frequently implicated in diabetic wounds. To ascertain the presence of multiple antibiotic resistance in bacterial pathogens derived from diabetic wound infections, a comprehensive analysis is required.

Materials and methods: The present cross-sectional investigation was carried out at a tertiary care facility. The samples were collected in aseptic conditions from the Endocrinology unit, specifically from local in-hospital patients (n=140). These samples were then assessed for their susceptibility to the commonly used antibacterial medications within the study area. The specimens were obtained from the lesions of individuals diagnosed with diabetes. The subjects were subjected to inoculation using various media and cultures.

Results: The findings of this study revealed that a collective sum of 122 bacterial isolates was acquired. The conclusions of the antibiotic susceptibility analysis revealed that the gram-positive isolates had a higher level of resistance to penicillin G (93.18%). However, they demonstrated sensitivity to vancomycin (100%) and linezolid (LZD) (95%). The gram-negative isolates exhibited complete resistance, at a rate of 100%, to penicillin, specifically amoxicillin (AMC), as well as to sulfonamides, such as sulfamethoxazole/trimethoprim (SXT), which belong to the antibiotic classes mentioned.

Conclusion: In conclusion, there has been a notable rise in antibiotic resistance.

## Introduction

Diabetes mellitus is a persistent metabolic disorder distinguished by heightened blood glucose, also known as blood sugar. Over time, the condition significantly harms several bodily organs, including but not limited to the heart, blood vessels, eyes, kidneys, and nerves [1]. Infected wounds are a significant consequence commonly observed in individuals with diabetes. Minor injuries are an inevitable and distressing facet of human existence. Nevertheless, these injuries can lead to substantial health complications among individuals diagnosed with diabetes. The individuals in question have delayed wound healing due to hyperglycemia, impaired blood circulation, neuropathy, and compromised immunological function. Based on data provided by the World Health Organization, it is evident that the prevalence of diabetes mellitus has shown a gradual increase over time. In 1980, over 108 million individuals were affected by this condition. The global prevalence of diabetes exhibited an upward trend, with the number of diabetic patients rising from 151 million in 2000 to 194 million in 2003, 246 million in 2006, 285 million in 2009, 366 million in 2011, and 425 million in 2015 [2]. According to recent data, the global prevalence of diabetes in 2021 is estimated at approximately 537 million individuals. Projections indicate that this figure is anticipated to rise to 643 million by 2030 and further increase to 783 million by 2045 [3].

Diabetes foot ulcers (DFUs) are estimated to impact approximately 10%-15% of those with diabetes at some point. At the time of presentation, it has been shown that roughly 50% of diabetic foot ulcers (DFUs) exhibit clinical signs of infection. *Staphylococcus aureus *and beta-hemolytic Streptococci are the two primary etiological agents responsible for skin infections. In contrast, gram-negative bacteria, including *Pseudomonas aeruginosa*, are more prevalent in nations with fewer resources. It has been documented that fungi can infect wounds in individuals with diabetes [4]. Bacterial strains obtained from the wounds of individuals with diabetes exhibit various types, encompassing gram-positive and gram-negative bacteria. The bacterial species that fall within the *Staphylococcus* genus are *S. aureus* and *Staphylococcus epidermidis*. Similarly, the *Streptococcus* genus contains *Streptococcus agalactiae*, *Streptococcus pyogenes*, and *Streptococcus mitis*. The *Enterococcus* genus includes *Enterococcus faecalis*, while the Enterobacteriaceae family comprises *Escherichia coli*, *Klebsiella*, and *Proteus mirabilis*. In addition, previous studies have identified the presence of Prevotella, Clostridium species, Aerococcus, and Halococcus [4]. A survey conducted in Kenya showed that 94% of the swabs collected from the wounds of individuals with diabetes yielded positive results when subjected to culture analysis. Among these positive results, 29% were identified as gram-positive bacteria, while 65% were identified as gram-negative. The predominant microorganisms identified in the study were *S. aureus* (16%), *E. coli* (15%), *P. mirabilis* (11%), *Klebsiella pneumoniae* (7%), and *P. aeruginosa* (7%).

The findings of a study conducted at a tertiary care hospital in Pakistan revealed that piperacillin/tazobactam was found to be an effective antibiotic against the most frequently encountered species in diabetic foot ulcer (DFU) infections, namely non-*S. aureus* (35.48%), *P. aeruginosa* (22.26%), and *S. aureus* (20.96%) [5]. The emergence of antimicrobial resistance (AMR) is becoming recognized as a significant global concern. The identification of methicillin-resistant *Staphylococcus aureus* (MRSA) dates back to the early 1960s, its association with prolonged hospitalization increased healthcare expenditures, and elevated mortality rates have been established. A study conducted in Kenya revealed that a significant proportion of bacterial isolates obtained from diabetic foot samples exhibited resistance to various antibiotics, including ampicillin, amoxicillin, cefepime, ceftazidime, cefuroxime, clindamycin, erythromycin, piperacillin-tazobactam, tetracycline, and trimethoprim-sulfamethoxazole. The presence of multidrug-resistant organisms was observed in 31% of the isolates of *S. aureus* and 40% of the gram-negative isolates. In the context of studies conducted in Morocco, it was observed that methicillin-resistant *Staphylococcus aureus* (MRSA) constituted approximately 4.7% of the total *S. aureus* isolates. The prevalence of vancomycin resistance in methicillin-resistant *Staphylococcus aureus* (MRSA) infections in Brazil was 33%. Multidrug-resistant organisms (MDROs) refer to microorganisms that exhibit resistance to various kinds of antibiotics. The results of antibiotic susceptibility testing (AST) conducted on bacterial isolates from diabetic foot ulcers (DFUs) in Tanzania revealed a noteworthy prevalence of antimicrobial resistance (AMR) [6]. The objective of our study is to ascertain distinct bacterial isolates present in each sample, evaluate the minimum inhibitory concentration (MIC) of multidrug-resistant isolates, and determine the genetic factors responsible for drug resistance in multidrug-resistant (MDR) bacterial strains.

## Materials and methods

Methodology

The design of the study and the duration of the study period were determined and implemented under established research methodologies. The present investigation was a cross-sectional, multi-sectoral study between November 2019 and March 2020, approved by the Department of Medical Research, Rehman Medical College with approval number Q-498045.

The Compilation of Specimens

The wound samples from diabetes patients were collected at Hayatabad Medical Complex Peshawar, a Medical Teaching Institution. These samples were taken using sterile syringes or pure cotton swabs and transported to the Microbiology laboratory. Upon arrival, the samples were stored at a temperature of 4°C for future use.

The Process of Isolating Pathogenic Bacteria

The specimens were introduced onto blood agar media, mannitol salt agar (MSA), and MacConkey agar media obtained from individuals with diabetes using a sterile wire loop. Subsequently, they were placed in an incubator at a temperature of 37°C for an overnight duration. The process of morphological identification involved the examination of colonies that were pure and isolated.

Identification of Bacterial Cultures

Morphological characteristics of pure bacterial cultures, including their color, size, growth patterns, and odor, were examined. Additionally, the bacterial colonies exhibited variations in density, lactose fermentation capability, suspension levels, and hemolytic activity. The findings were subsequently recorded. Gram staining and biochemical tests, including catalase, oxidase, coagulase, etc., were conducted according to established protocols to get preliminary identification data on pathogenic bacteria.

The Gram Staining Technique

The gram staining technique was employed to discern and distinguish the bacterial colonies based on their gram-positive or gram-negative characteristics. The present study aims to conduct a biochemical characterization of the subject under investigation. To forward the process of identification, the isolated colonies underwent additional screening utilizing a range of biochemical tests, including oxidase, indole, catalase, urease, citrate, coagulase, Triple Sugar Iron (TSI), and Triple Sugar Iron with Slant and Butt (TSI).

The Preservation of Bacterial Cultures

The slants were made using nutrient agar, and the pure cultures were inoculated onto the slants. Subsequently, the slants were incubated at 37°C for one night. The slants were afterward stored at a temperature of 4°C in a refrigeration unit. The method employed for disc diffusion analysis is widely used in microbiology to assess the antimicrobial activity of various substances. The Kirby-Bauer disc diffusion method was employed to evaluate the susceptibility of each bacterial isolate, using Mueller-Hinton agar as the culture medium. Following this methodology, a filter paper was immersed in a solution of antibiotics with a predetermined concentration. The organism to be evaluated for sensitivity to the antibiotic is introduced into the media used for cultivation and analysis. The antibiotics undergo diffusion within the medium, inhibiting bacterial growth. The media preparation process adhered to the established protocols. The media was prepared according to established procedures, subjected to autoclaving, and incubated at 37°C for 24 hours to assess the sterility of the plates [4].

Antibacterial Sensitivity Assay

The antibacterial sensitivity testing was conducted on the isolated bacterial cultures using clinically effective antibiotics. The efficacy of each antibiotic against each isolate was determined based on the guidelines provided by the Clinical and Laboratory Standards Institute (CLSI) 2012 [5], as presented in Table 1.

**Table 1:** Antibacterial agents and their sensitivity

Antibacterial drugs	Resistant (mm)	Sensitivity (mm)	Intermediate (mm)
CIP (ciprofloxacin)	≤15	≥2	16-19
IMP (imipenem)	≤13	≥17	14-16
FEP (cefepime)	≤13	≥18	14-17
AMC (ampicillin)	≤12	≥17	13-16
TZP (tazobactam/piperacillin)	≤16	≥21	17-20
CRO (ceftriaxone)	≤15	≥23	16-22
CAZ (ceftazidime)	≤13	≥17	14-16
DOX (doxycycline)	≤12	≥17	13-16
CN (gentacin)	≤11	≥14	12-13
POL-B (polymyxin B)	≤12	≥16	13-15
SCF (cefoperazone)	≤14	≥21	15-19
MEM (meropenem)	≤12	≥16	13-15
AK (amikacin)	≤14	≥18	15-16
ATM (aztreonam)	≤15	≥21	16-20
LEV (levofloxacin)	≤13	≥18	14-17
CTX (cefotaxime)	≤14	≥22	15-21

The Process of Preparing the Inoculum

In this study, an ampoule of sterile distilled water that is commercially available was utilized for the preparation of inoculums. The bacterial inoculants with hazardous properties were standardized to a concentration of 0.5 McFarland units. A sterilized cotton swab was immersed into a standardized bacterial suspension. The interior walls of the tubes were gently squeezed using a sterile cotton swab in order to acquire an ample amount of culture. The Mueller-Hinton agar was evenly spread using a cotton swab in three directions, resulting in uniform and reliable growth. The antibacterial medicines (discs) of established concentrations were applied to the media surface after a 15-minute incubation period following injection using a disc dispenser. The plates were subjected to overnight incubation at 37°C, with the plates positioned in an inverted manner. Following the incubation period, the measurement of inhibition zones was conducted.

The Minimum Inhibitory Concentration (MIC)

The minimum inhibitory concentration (MIC) refers to the concentration of antibiotics that completely inhibits microbial growth following an incubation period of one night. The primary objective of the agar and broth dilution procedure was to ascertain the minimum concentration of the tested antibacterial medications that effectively suppress the observable growth of the studied bacterium, within the specified experimental parameters. The significance of determining the minimum inhibitory concentration (MIC) lies in its ability to ascertain the sensitivity of microorganisms to pharmaceutical agents and evaluate the efficacy of novel antibacterial compounds. The process of agar dilution entails the incorporation of various quantities of antibacterial agents into the N-agar medium (nutrient), which is subsequently spread evenly throughout the surface of an agar plate using a standardized technique. Frequently, to employ the broth dilution approach using a 96-well microtiter plate format, microorganisms that have been infected are introduced into a liquid growth medium with varying quantities of antibacterial medication. The growth was assessed during incubation for 18-24 hours, and the minimal inhibitory concentration (MIC) value was determined. This approach applies to aerobic microorganisms and is typically conducted within three days [6].

Preparation of Antibacterial Agents

The antibacterial medicines were dissolved in water and introduced into a molten agar medium. A solution of distilled water (dH_2_O) with a concentration of 10× was created to dilute antibacterial drugs. The minimal inhibitory concentration (MIC) was shown to vary across different medications. In accordance with the recommendations established by the Clinical and Laboratory Standards Institute (CLSI) in 2012, a range of minimum inhibitory concentrations (MICs) were adhered to.

Preparations for Plates

The Mueller-Hinton agar medium was sterilized by autoclaving in 100 ml flasks and afterward cooled in a water bath set at 50°C. The intermediate antibiotics were added to each flask at a concentration of 10 times the desired final concentration in the appropriate volume. The mixture was then carefully combined and immediately poured onto each plate holding the antibacterial medications. Antibiotics were incorporated into the agar medium using a two-fold serial dilution technique. The antibiotic plates were prepared with varying concentrations of 50 μg/ml, 100 μg/ml, 250 μg/ml, 500 μg/ml, and 1000 μg/ml. The test microorganism was acquired by inoculating agar from an overnight culture. A minimum inhibitory concentration test was conducted using an inoculum from three to five distinct and morphologically similar colonies obtained from an agar plate culture. The upper portion of each colony was aseptically collected using a sterile wire loop and transferred into a tube containing 0.4-0.5 ml of standard saline solution without any microbial contamination. The culture broth was incubated at 35°C for a duration typically ranging from two to six hours until it reached the desired turbidity level according to McFarland standards, namely a turbidity of 0.5. The culture broth turbidity was established by inoculating germ-free broth to attain a turbidity level similar to McFarland standards (0.5). The process of incubation and injection of the medium involves the placement of a substance in a controlled environment to facilitate its growth or development, followed by the introduction of another substance into the medium by a specific method or technique. The control plate was spot inoculated with a suspension of 0.2 μl without antibacterial medications using a digital micropipette. The agar media plates contained varying amounts of antibacterial pharmaceuticals. The plates composed of the lowest concentration of antibiotics were utilized, and the control plate was afterward infected. The infected leaves were incubated overnight at 37°C until the inoculum spot was completely absorbed.

The Identification of Multidrug-Resistant Isolates

Multidrug resistance was designated to isolates that exhibited resistance to a minimum of three distinct classes of antibiotics [7]. The microorganisms that were in isolation were subjected to a screening process to identify multidrug-resistant (MDR) isolates. Subsequently, the identified MDR isolates were appropriately labeled. The phenomenon of molecular resistance refers to the ability of organisms to develop mechanisms that render them less susceptible to the effects of specific molecules. The identification and characterization of genes were extracted. DNA extraction was conducted subsequent to a phenotypic investigation to detect multidrug-resistant (MDR) genes among the bacterial isolates. The DNA extraction from multidrug-resistant (MDR) isolates was performed using the usual phenol-chloroform procedure, as described in a previous study [8]. The experiment commenced by incubating fresh broth cultures for 24 hours. Subsequently, 1.5 ml of the inoculum was placed into a broth culture and subjected to centrifugation for two minutes using sterile Eppendorf tubes. The liquid portion, known as the supernatant, was discarded. In contrast, the solid portion, referred to as the pellet, was reconstituted in a solution consisting of 570 units of Tris-EDTA (T.E.) buffer and 30 units of sodium dodecyl sulfates (SDS). After adding T.E. buffer and sodium dodecyl sulfate (SDS), the mixture should be incubated at 37°C for one hour. Subsequently, a mixture comprising 100 ml of 5 molar sodium chloride (NaCl) and 80 ml of cetyltrimethylammonium bromide (CTAB) in the presence of NaCl is subjected to incubation for 10 minutes within a water bath maintained at a temperature of 65°C. Equal volumes of phenol, chloroform, and isoamyl alcohol (P:C:I) were combined and centrifuged. The resulting top phase was carefully transferred into a new sterilized Eppendorf tube and centrifuged at 14,000 revolutions per minute (RPM) for five minutes. Next, a volume of isoamyl alcohol equal to 0.6 times the initial volume (750 * 0.6 = 450) was added, and the mixture was afterward stored at a temperature of -30°C for 30 minutes. The sample underwent a second round of centrifugation, resulting in the separation of the supernatant fraction. This separation was achieved by subjecting the sample to centrifugal forces of 14,000 revolutions per minute for three minutes. The pellet was supplemented with 100 T.E. buffer and subjected to overnight incubation.

Confirmation of DNA Extraction by Gel Electrophoresis

Before its utilization in molecular analysis, the DNA underwent extraction using gel electrophoresis. The agarose gel (0.1%) was produced using a 1x Tris-acetate-EDTA (TAE) buffer solution. The agarose was added in the amount of 0.8 g and dissolved in 80 ml of TAE buffer afterward. Agarose melting was conducted using a microwave oven, with a time interval of two to three minutes. The agarose was permitted to cool briefly, following which ethidium bromide was introduced. The agarose gel was carefully poured into a gel tray and allowed to harden for 20 to 30 minutes before introducing DNA samples into the tray. A solution of 6× loading dye was made by combining 0.25% xylene cyanol, 0.25% bromophenol blue, 30% glycerol, and an eight-fold diluted DNA sample. The gel tray was positioned onto the tank containing a solution of 1× TAE buffer. The wells created by the utilization of comb DNA samples were afterward filled with these samples. The gel tank has cathode and anode terminals with opposing positive and negative charges. These terminals are connected to a power supply with a voltage of 100 volts, and the system is allowed to operate for 20-30 minutes. Following the completion of electrophoresis, the gel was subjected to visualization utilizing the gel documentation system, commonly referred to as Gel Doc. The polymerase chain reaction (PCR) was employed to detect specific genes, namely *CTX*, *TEM*, and *OXA*. The polymerase chain reactions (PCRs) were conducted with a total volume of 25 µl in PCR tubes. The polymerase chain reaction (PCR) tube was composed of 12.5 µl of the master mix, 10.5 µl of PCR water, 0.5 µl each of the forward and reverse primers, and 0.1 µl of genomic DNA. The polymerase chain reaction (PCR) was conducted using the specified experimental conditions. The condition for polymerase chain reactions (PCRs) involves an initial denaturation step at 94°C for five minutes, followed by subsequent denaturation steps at 94°C for one minute. The annealing temperature was conducted at 58°C for one minute, while the extension temperature was at 72°C for one minute. The final extension phase was completed at a temperature of 72°C for a duration of five minutes. The stages mentioned above were executed in a total of 30 iterations. The process of generating primer stocks and the factors to consider for optimizing polymerase chain reactions (PCRs) are discussed. The utilization of specific gene primers was previously suggested. To provide further clarification, the conditions that were initially described were utilized. However, to obtain aesthetically pleasing products, these conditions did not yield superior outcomes, thus necessitating optimization techniques. Given this rationale, the annealing temperatures were established at 58°C, as delineated in Table 2.

**Table 2:** Target genes and their primers bp: base pair.

Target genes	Primer	DNA sequence (5´-3´)	Size of product (bp)	Annealing temperature (°C)
bla CTX-M-1	CTXM1-F CTXM1-R	CGTCACGCTGTTGTTAGGAA ACGCCTTTCTGCCTTAGGTT	499	58°C
bla TEM	TEM-F TEM-R	CTTCCTGTTTTTGCTCACC AGCAATAAACCAGCCAGC	516	58°C
bla OXA-1	OXA-F OXA-R	ATATCTCTACTGTTGCATCTCC AAACCCTTCAAACCATCC	619	58°C

Visualization of PCR Products

The polymerase chain reaction (PCR) was performed under the following conditions, as shown in Table 3.

**Table 3:** PCR condition PCR: polymerase chain reaction.

Denaturation		Annealing		Extension	
Temperature	Time interval	Temperature	Time interval	Temperature	Time Interval
94°C	5 minutes	58°C	1 minute	72°C	5 minutes

The PCR product was subjected to gel electrophoresis. The agarose gel with a concentration of 1.5% was produced using 1× TAE buffer for the intended purpose. The agarose was weighed at 1.2 g and subsequently dissolved in 80 ml of TAE solution. Agarose melting was conducted using a microwave oven, with a time interval of two to three minutes. The agarose was permitted to cool briefly, following which ethidium bromide was introduced into it. The agarose gel was carefully poured into a gel tray and allowed to set for a duration of 20 to 30 minutes, following which the DNA samples were placed into the tray. The experiment involved the addition of 6× loading dye, which was made by combining 0.25% xylene cyanol, 0.25% bromophenol blue, and 30% glycerol. Subsequently, a DNA sample was introduced into the mixture. The gel-containing tray was positioned onto the tank filled with a 1× TAE buffer solution. The wells created by the comb were subsequently filled with DNA samples. The gel tank is equipped with cathode and anode connections with positive and negative charges, which are concurrently connected to a 100-volt power supply for a duration of 20-30 minutes. Following the electrophoresis procedure, the Gel Doc system was employed to visualize the outcomes of the gel.

## Results

To screen out the pathogenic microorganisms, 140 specimens were collected from diabetic wound-infected patients. Among these samples, 122 samples yielded bacterial growth, which was further subjected to antibiotic sensitivity testing and identification.

Infection percentage on gender-wise

Among the 122 positive patients, 74 (60.70%) were male, while 48 (39.30%) were isolated from female participants, as shown in Figure 1.

**Figure 1:** Infection percentage in gender-wise distribution

Percentage of infections based on certain pathogens

All isolated bacteria were identified by utilizing gram staining response, colony morphology, and biochemical assays, with subsequent documentation of their respective percentages. In the dataset of 122 positive samples, *S. aureus* accounted for 36.90% of the isolates, *E. coli* accounted for 22.10%, *P. aeruginosa* accounted for 21.30%, *Enterobacter* spp. accounted for 5.70%, *Providencia* spp. accounted for 4.90%, *Proteus mirabilis* accounted for 4.80%, *Proteus vulgaris* accounted for 2.45%, and *Acinetobacter* accounted for 1.60%, as illustrated in Figure 2.

**Figure 2:** The percentage of infection with respect to pathogens

The percentage of infections categorized by age

The participants included individuals ranging in age from one to 90 years. The individuals were categorized into four distinct age groups, as depicted in Figure 3.

**Figure 3:** Percentage of infection with respect to the age of patients

Within the age range of 41-60 years, a higher proportion of samples (37.70%) were isolated, whereas a lower proportion of samples (17.21%) were isolated from patients above 60 years. The number of patients aged one to 20 years experienced a reduction of 18.03%. The age group of 21-40 years had a significant prevalence of microorganisms, accounting for 27.04% of the total sample.

The antibiotic susceptibility profile of isolated bacteria

A total of 13 to 16 antibiotics were employed in this study for each isolate, with consideration given to the diverse classes of antibiotics. The antibiotics were chosen from various antibiotic classes, such as cephalosporin, carbapenem, aminoglycosides, penicillin, fluoroquinolones, polymyxin B, and tetracycline.

Determination of multidrug-resistant (MDR) status with respect to gender

This investigation revealed 36 multidrug-resistant (MDR) isolates, accounting for 29.50% of the sample. Among these isolates, 24 were obtained from male and 12 from female patients. The distribution of these isolates across different age groups is presented in Table 4. 

**Table 4:** Number of isolated multidrug-resistant (MDR) pathogens in male and female patients

Gender	Number and percentage of patients	Age grouping	MDR isolates number and percentage
Male	24 (66.66%)	1-20 years	2 (5.5%)
		21-40 years	5 (13.88%)
		41-60 years	10 (27.77%)
		Above 60 years	7 (19.44%)
Female	12 (33.33%)	1-20 years	1 (2.77%)
		21-40 years	7 (19.44%)
		41-60 years	3 (8.33%)
		Above 60 years	0
Total	36 (100%)		

Figure 4 demonstrates that 26 isolates of *P. aeruginosa* exhibited complete resistance, amounting to 100%, to penicillin antibiotics such as amoxicillin (AMC) and sulfonamides such as sulfamethoxazole/trimethoprim (SXT). Out of the 26 samples of *P. aeruginosa* that were examined, it was shown that the resistance rate to tazobactam/piperacillin (TZP) was 13.33%, while the susceptibility rate was 86.67%. The group of antibiotics known as cephalosporin, namely cefotaxime (CTX) and ceftriaxone (CRO), exhibited resistance rates of 60% and 6.67%, respectively. Conversely, susceptibility rates to these medications were 26.67% and 53.33%, with intermediate resistance rates at 13.3% and 40%, respectively. In the context of sulbactam/cefoperazone, a combination of a third-generation cephalosporin and a β-lactamase inhibitor, the sensitivity was 93.33%. In comparison, the resistivity was reported to be 6.67%. In ceftazidime (CAZ), 73.33% of the samples exhibited susceptibility, while 27.67% showed resistance. Polymyxin E, also known as colistin sulfate (CT), had a sensitivity rate of 100% against *P. aeruginosa* isolates. On the other hand, polymyxin B (PB) demonstrated susceptibility in 86.67% of cases, while 13.33% of the isolates displayed resistance. The fluoroquinolone ciprofloxacin (CIP) was used to treat all samples of *P. aeruginosa*. The sensitivity of ciprofloxacin was determined to be 53.33%, while the resistance rate was 33.33%. Additionally, an intermediate response was observed in 13.33% of the samples. Amikacin (AK), belonging to the aminoglycosides group, was administered against all samples of *P. aeruginosa*. The sensitivity of this treatment was determined to be 86.67%, while the resistivity was found to be 13.33%. Tetracycline drugs, specifically minocycline (MH) and clindamycin (DA), a derivative of lincomycin, exhibited resistance rates of 73.33% and 46.67%, respectively. The sensitivity rates for both antibiotics were 20% and 53.33%. A 6.67% intermediate resistance was explicitly determined for minocycline (MH).

**Figure 4:** Potency of various antibiotics against Pseudomonas aeruginosa AMC: ampicillin, CIP: ciprofloxacin, CTX: cefotaxime, TZP: tazobactam/piperacillin, CAZ: ceftazidime, SCF: cefoperazone, CRO: ceftriaxone, PB: polymyxin B, MH: minocycline, AK: amikacin, CT: cefotaxime, DA: clindamycin, SXT: trimethoprim/sulfamethoxazole.

Figure 5 illustrates that among the 45 *S. aureus* isolates, 95% exhibited sensitivity to the penicillin group of antibiotics, specifically amoxicillin (AMC), while 5% were classified as resistant. In contrast, the sulfonamides group of antibiotics, including sulfamethoxazole/trimethoprim (SXT), demonstrated a resistance rate of 63%, with 37% of isolates being susceptible. The study observed that 45 *S. aureus* isolates had a sensitivity rate of 43% to piperacillin/tazobactam (TZP), with a resistance rate of 25%. Additionally, 32% of the isolates demonstrated intermediate resistance.

**Figure 5:** Antibiotic sensitivity pattern of Staphylococcus aureus to various antibiotics AMC: ampicillin, CIP: ciprofloxacin, CTX: cefotaxime, TZP: tazobactam/piperacillin, CAZ: ceftazidime, SCF: cefoperazone, CRO: ceftriaxone, VA: vancomycin, CN: cefalexin, P: penicillin G, DA: clindamycin, LZD: linezolid, RD: metronidazole, E: erythromycin, DO: doxycycline, SXT: trimethoprim/sulfamethoxazole.

The susceptibility of the cephalosporin cefotaxime (CTX) was 52%, with resistance observed in 16% of cases and intermediate resistance in 32% of cases. Similarly, ceftriaxone (CRO) exhibited a sensitivity rate of 45%, a percentage resistance rate of 18%, and a percentage intermediate resistance rate of 36%. The combination of sulbactam and cefoperazone (SCF), which consists of a third-generation cephalosporin inhibitor and β-lactamase, exhibited a sensitivity rate of 48%. The resistivity rate was 23%, while 29% of cases demonstrated intermediate resistance. In the case of ceftazidime (CAZ), 50% of patients were susceptible, 16% exhibited resistance, and 34% showed intermediate resistance. Penicillin G (P) had a resistance rate of 93%, but its sensitivity rate was 7%. Gentamicin, a member of the aminoglycoside class of antibiotics, exhibited a susceptibility rate of 75%. The resistivity rate was 23%, while 2% of cases were classified as demonstrating intermediate resistance. Linezolid (LZD), belonging to the oxazolidinone class of antibiotics, had a susceptibility rate of 95%, with 2% of cases demonstrating resistance or intermediate levels of susceptibility. Rifampicin (RD) is classified as a member of the complex macrocyclic group of antibiotics. It has been observed to exhibit a sensitivity rate of 86%, while its resistivity rate is recorded at 11%. Additionally, an intermediate resistance rate of 3% has been determined. Clindamycin, a derivative of lincomycin antibiotics, exhibited a sensitivity rate of 75%, a resistance rate of 20%, and an intermediate rate of 5%. The fluoroquinolone ciprofloxacin (CIP) was administered to all samples of *S. aureus*. The resistivity of ciprofloxacin was determined to be 43%, with a sensitivity of 34% and 23% exhibiting intermediate resistance.

The glycopeptide antibiotic vancomycin (VA) was employed to combat all strains of *S. aureus*, with a sensitivity rate of 100% being determined. Tetracycline antibiotics, including doxycycline (DO), and macrolides antibiotics, such as erythromycin (E), were found to have a sensitivity rate of 93% and a resistance rate of 5%, with 2% classified as intermediate resistance. Similarly, erythromycin (E) from the macrolides class of antibiotics exhibited a sensitivity rate of 52%, a resistance rate of 43%, and 5% were classified as intermediate resistance.

The data presented in Figure 6 indicates that out of the 27 *E. coli* isolates examined, 54% exhibited resistance to penicillin, specifically amoxicillin (AMC). Conversely, 46% of the isolates were susceptible to this antibiotic. In terms of the sulfonamides group of antibiotics, namely sulfamethoxazole/trimethoprim (SXT), 77% of the isolates displayed resistance, while 23% were classified as sensitive. The susceptibility of tazobactam/piperacillin (TZP) was 85% among 28 *E. coli* samples. The resistivity rate was 7%, while 6% of the samples were classified as intermediate. The group of antibiotics known as cephalosporin, specifically cefotaxime (CTX) and ceftriaxone (CRO), exhibited resistance rates of 77% and 38%, respectively. Conversely, susceptibility rates to these medications were 8% and 31%, while intermediate resistance was observed at 15% and 31%. The combination of sulbactam/cefoperazone (SCF) is a third-generation cephalosporin inhibitor and β-lactamase with a sensitivity rate of 85%. The rates of resistance and intermediate resistance were 7% and 6%, respectively. In the case of ceftazidime (CAZ), 62% of patients were classified as resistant, 31% as susceptible, and 7% as intermediate resistance.

**Figure 6:** The sensitivity pattern of Escherichia coli to various antibiotics AMC: ampicillin, CIP: ciprofloxacin, CTX: cefotaxime, TZP: tazobactam/piperacillin, CAZ: ceftazidime, SCF: cefoperazone, CRO: ceftriaxone, PB: polymyxin B, MH: minocycline, AK: amikacin, CT: cefotaxime, DA: clindamycin, SXT: trimethoprim/sulfamethoxazole.

Polymyxin E, colistin sulfate (CT), and polymyxin B (PB) demonstrated a sensitivity rate of 100% when tested against *E. coli* isolates. The fluoroquinolone ciprofloxacin (CIP) was administered to all samples of *E. coli*. The resistivity of ciprofloxacin was determined to be 69%, whereas 31% of the samples were found to be sensitive. Amikacin (AK), a member of the aminoglycosides group, was administered to all *E. coli *samples to evaluate its efficacy. The sensitivity of AK was determined to be 92%, while the resistance rate was found to be 8%. Tetracycline antibiotics, specifically minocycline (MH) and clindamycin (DA), a derivative of lincomycin, exhibited resistance rates of 39% and 62%, respectively. The sensitivity rates for both antibiotics were 23% and 38%. Additionally, the intermediate resistance rate for minocycline (MH) was assessed to be 38%.

MDR isolates

The data shown in Figure 7 demonstrates that out of the total MDR isolates, 36 exhibited a resistivity of 97% toward penicillin, specifically amoxicillin (AMC), whereas 3% had intermediate resistance. Furthermore, the sulfonamides group of antibiotics, such as sulfamethoxazole/trimethoprim (SXT), demonstrated a resistivity of 100%. The study observed that among the 36 multidrug-resistant (MDR) samples, the resistance rate to piperacillin/tazobactam (TZP) was 68%. Conversely, the susceptibility rate was 22%, while 11% of the samples exhibited intermediate resistance. The isolates exhibited a resistivity of 90% to cephalosporin/cefotaxime (CTX), with no detected susceptibility. However, 0.3% of the isolates demonstrated intermediate resistance. In contrast, all isolates displayed 100% resistance to ceftriaxone (CRO). The combination of sulbactam/cefoperazone (SCF), which consists of a β-lactamase inhibitor and a third-generation cephalosporin, exhibited a resistance rate of 53%. Sensitivity rates were 31%, while 16% showed intermediate resistance. In ceftazidime (CAZ), 86% of cases were classified as resistant, while 14% were found to be susceptible. The isolates exhibited a sensitivity rate of 75% when exposed to polymyxin E, also known as colistin sulfate (CT), and a susceptibility rate of 79% when exposed to polymyxin B (PB). The resistance rate for colistin sulfate (CT) isolates was 25%, while 22% exhibited intermediate resistance to polymyxin B (PB). The fluoroquinolone ciprofloxacin (CIP) was administered to all samples with multidrug resistance (MDR). Among these samples, 89% exhibited resistance to ciprofloxacin, while 8% displayed sensitivity to the drug. Only 3% of the samples demonstrated intermediate resistance. Amikacin (AK), a member of the aminoglycosides group, was administered to combat all multidrug-resistant (MDR) samples. The resistivity rate was 72%, indicating a high resistance level. Conversely, the susceptibility rate was found to be 25%, indicating a relatively low level of effectiveness. Additionally, 3% of the samples were classified as exhibiting intermediate resistance. Tetracyclines, including minocycline (MH) and clindamycin (DA), derivatives of lincomycin antibiotics, exhibited a resistance rate of 56%. Conversely, a sensitivity rate of 25% was explicitly seen for minocycline (MH). Nineteen percent of the samples exhibited moderate resistance. In opposition to linezolid (LZD), a member of the oxazolidinone class, it was observed that 78% of isolates exhibited resistance, 19% demonstrated intermediate resistance, and 3% displayed sensitivity. Vancomycin (VA), an antibiotic from the glycopeptides class, was administered to combat multidrug-resistant (MDR) isolates. Among these isolates, 83% exhibited resistance to vancomycin, while the remaining 3% were found to be sensitive, and 16% had intermediate resistance.

**Figure 7:** The sensitivity pattern of multidrug-resistant (MDR) isolates against various antibiotics AMC: ampicillin, CIP: ciprofloxacin, CTX: cefotaxime, TZP: tazobactam/piperacillin, CAZ: ceftazidime, SCF: cefoperazone, CRO: ceftriaxone, PB: polymyxin B, MH: minocycline, AK: amikacin, CT: cefotaxime, DA: clindamycin, SXT: trimethoprim/sulfamethoxazole, LZD: linezolid, VA: vancomycin, MEM: meropenem.

Multidrug resistance among isolated pathogens

Isolates that exhibit resistance to a minimum of three types of antibiotics will be classified as multidrug-resistant (MDR). Thirty-six isolates were found to belong to this category, as indicated in Table 5.

**Table 5:** Multidrug resistance isolates among 122 isolates

S. No	Group I	Group II	Group III	Group IV	Group V
1	Penicillin	Aminoglycoside	Cephalosporin		Sulfonamide
2	Penicillin		Cephalosporin	Fluoroquinolone	Sulfonamide
3	Penicillin	Aminoglycoside	Cephalosporin	Fluoroquinolone	
4	Penicillin	Aminoglycoside	Cephalosporin		Carbapenem
5	Penicillin	Aminoglycoside	Cephalosporin	Fluoroquinolone	
6		Aminoglycoside	Cephalosporin		Tetracycline
7	Penicillin	Aminoglycoside	Cephalosporin	Fluoroquinolone	
8	Penicillin	Aminoglycoside	Cephalosporin		Polymyxin B
9	Penicillin	Aminoglycoside	Cephalosporin	Fluoroquinolone	
10	Penicillin	Aminoglycoside	Cephalosporin		Sulfonamide
11	Penicillin			Fluoroquinolone	Tetracycline
12		Aminoglycoside		Fluoroquinolone	Tetracycline
13	Penicillin	Aminoglycoside		Fluoroquinolone	
14		Aminoglycoside	Cephalosporin		Tetracycline
15	Penicillin		Cephalosporin	Fluoroquinolone	
16	Penicillin	Aminoglycoside	Cephalosporin	Fluoroquinolone	
17		Aminoglycoside		Fluoroquinolone	Carbapenem
18	Penicillin		Cephalosporin	Fluoroquinolone	
19	Penicillin		Cephalosporin	Fluoroquinolone	Polymyxin B
20	Penicillin		Cephalosporin	Fluoroquinolone	Tetracycline
21	Penicillin	Aminoglycosides	Cephalosporin	Fluoroquinolone	
22	Penicillin		Cephalosporin	Fluoroquinolone	Polymyxin B
23	Penicillin	Aminoglycosides	Cephalosporin	Fluoroquinolone	
24	Penicillin	Aminoglycosides	Cephalosporin	Fluoroquinolone	
25	Penicillin		Cephalosporin	Fluoroquinolone	
26	Penicillin	Aminoglycosides	Cephalosporin	Fluoroquinolone	
27	Penicillin		Cephalosporin	Fluoroquinolone	
28	Penicillin	Aminoglycosides	Cephalosporin		Polymyxin B
29	Penicillin		Cephalosporin	Fluoroquinolone	
30	Penicillin	Aminoglycosides	Cephalosporin	Fluoroquinolone	
31	Penicillin		Cephalosporin	Fluoroquinolone	
32	Penicillin		Cephalosporin	Fluoroquinolone	
33	Penicillin	Aminoglycosides	Cephalosporin		
34	Penicillin		Cephalosporin	Fluoroquinolone	
35	Penicillin		Cephalosporin	Fluoroquinolone	
36	Penicillin	Aminoglycosides	Cephalosporin	Fluoroquinolone	

Table 6 presents a comprehensive statistical analysis of the drugs administered to patients with diabetes-related wounds, explicitly focusing on multidrug-resistant (MDR) isolates. The study categorizes the drugs based on their susceptibility to the MDR isolates, with a numerical representation: 1 for susceptible, 2 for intermediate, and 3 for resistant.

**Table 6:** Antibiotic sensitivity of multidrug-resistant isolates AMC: ampicillin, CIP: ciprofloxacin, CTX: cefotaxime, TZP: tazobactam/piperacillin, CAZ: ceftazidime, SCF: cefoperazone, CRO: ceftriaxone, PB: polymyxin B, MH: minocycline, AK: amikacin, CT: cefotaxime, DA: clindamycin, SXT: trimethoprim/sulfamethoxazole, VA: vancomycin, CN: cefalexin, P: penicillin G.

Antibiotics	MDR Isolates		
	Susceptible	Intermediate	Resistant
AMC	49.2	1.6	49.2
CIP	29.5	13.1	57.4
CTX	29.5	16.4	54.1
TZP	53.3	15.6	31.1
CAZ	43.4	13.9	42.6
SCF	58.2	16.4	25.4
CRO	35.2	21.3	43.4
PB	91.8		8.2
MH	45.1	14.8	40.2
AK	41.8	0.8	57.4
CT	83.6	1.6	14.8
DA	49.2	0.8	50
SXT	33.6	0.8	65.6
VA	52.3	4.5	43.2
CN	93.2	2.3	4.5
P	36.4		63.6

Result analysis

The minimum inhibitory concentration (MIC) refers to the concentration of antibiotics that completely suppresses microbial growth following an incubation period of one night. The final data points, which consisted of barely perceptible or solitary growth colonies, were disregarded. The results were computed based on the CLSI 2012 reference chart. Regarding the minimum inhibitory concentration concept, the antibiotics tested and administered strains are denoted as resistant (R) and susceptible (S). The minimum inhibitory concentration (MIC) values for *E. coli*, including isolates digital karyotyping (DK) 01 and DK 02, indicated a high resistance level to the antibiotics tested, namely CRO and AMC. Notably, proliferation was seen even at the highest concentration of 1000 µg/ml. The isolate number DK 05 was exclusively detected at the tested dose concentrations of 250, 500, and 1000 µg/ml. The minimum inhibitory concentration (MIC) values for *S. aureus* were determined. The results indicated that growth was only found at the highest concentration of 1000 µg/ml^-1^ among the five isolates tested, specifically isolate number DK. The growth of isolate numbers DKW, DK 04, DK 09, and DK10 was assessed in terms of milliliters against LZD, VA, and AMC. However, when tested against SEP, MXP, and levofloxacin (LEV), the growth was detected at 1000 µg/ml concentration. Isolate number 50 exhibited resistance to fosfomycin (FOS) ciprofloxacin (CIP), MXP, and enoxacin (ENX), with no apparent growth reduction. The MIC values for *Enterobacter* and *Pseudomonas* species were determined. Among the *Enterobacter* species, isolate 70 exhibited the highest MIC values, indicating no growth at the highest concentration of antibiotics tested. Isolate 41 resisted gentamicin (GEN), sulfonamides (SUL), meropenem (MEM), triglyceride and glucose index (TYG), and cefepime (CEF) antibiotics. In contrast, isolate number 60 of the *Enterobacter* species demonstrated minimum inhibitory concentration (MIC) values between 500 and 1000 µg/ml^-1^ against several antibiotics. The isolate number 90 exhibited resistance to antibiotics such as GEN, FOS, and CIP, as evidenced by its unhindered growth even at a concentration of 1000 µg/ml. The minimum inhibitory concentration (MIC) values for various species of *Pseudomonas* were determined. The minimum inhibitory concentration (MIC) values of *Pseudomonas* isolates DK 02 and DK 05 indicated that their growth was solely seen when exposed to ciprofloxacin (CIP) and ceftriaxone (CRO) at a concentration of 1000 µg/ml. The MIC values of the tested substance against meropenem (MEM) and SCF were observed to be 250, 500, and 1000 µg/ml.

Molecular characterization

Following phenotypic verification, the bacterial isolates underwent additional processing for molecular characterization to identify multidrug-resistant (MDR) isolates through the amplification of *bla CTX-M-1* and *bla TEM* genes.

Extraction of genomic DNA and analysis of results

The DNA was extracted from multidrug-resistant (MDR) isolates using the usual phenol-chloroform technique. The DNA was subjected to agarose gel electrophoresis with a concentration of 0.1%. The resulting bands were observed and documented using Gel Documentation.

Analysis of the product by gel electrophoresis

A total of 36 clinical isolates exhibiting multidrug resistance (MDR) were obtained from patients with infected diabetic wounds during the designated study period. The gel electrophoresis approach was employed to visually confirm the presence of *bla CTX-M-1* gene bands in polymerase chain reaction (PCR) detection of *P. aeruginosa*. The *bla CTX-M-1* gene bands of *P. aeruginosa*, which were isolated from 36 multidrug-resistant (MDR) isolates, were successfully created with a predictable size of around 499 base pairs (bps), as illustrated in Figures 8, 9.

**Figure 8:** Gene detection: bands of (499 bp) corresponding to the amplified region bla CTX-M-1 M=50-1000 bp DNA ladder, 10th, 16th, and 18th *Pseudomonas aeruginosa* isolates. bp: base pair.

**Figure 9:** Gene detection: bands of (516 bp) corresponding to the amplified region bla TEM gene M=50-1000 bp DNA ladder, eighth, and fourth *Escherichia coli* isolates. bp: base pair.

The plasmid DNAs were recovered from multidrug-resistant (MDR) isolates of *E. coli* that may exhibit extended-spectrum beta-lactamase (ESBL) activity. PCR *bla TEM*-specific primers were used to screen all ESBLs. The TEM PCR products were sequenced sequentially and compared to DNA Gen Bank sequences using a Basic Local Alignment Search Tool (BLAST) search. Extended-spectrum beta-lactamases (ESBLs) were predominantly detected in isolates of *E. coli*, although none of the isolates exhibited the presence of *bla OXA* genes. The prevalence of extended-spectrum beta-lactamase (ESBL) genes in *E. coli* was predominantly observed in the *bla TEM* gene variant. In recent years, there has been a progressive rise in global challenges about the growing resistance of pathogens to antibacterial medications, posing significant threats to public health. Numerous bacterial species, predominantly belonging to the Enterobacteriaceae family, can produce β-lactamase enzymes. These enzymes play a crucial role in the hydrolysis and subsequent inactivation of β-lactam antibiotics, making them a significant resistance mechanism. The prevalence of resistance to extended-spectrum β-lactams (ESBLs) in gram-negative organisms is progressively linked to the presence of ESBLs. Most enterobacterial species positive for extended-spectrum beta-lactamase (ESBL) are increasing globally.

## Discussion

This investigation aimed to perform molecular characterization and assess the sensitivity pattern of antibacterial medications for microbial strains isolated from individuals with diabetic wounds. The present study demonstrates that numerous organisms are responsible for producing infections in individuals with diabetes, with the most frequent and severe pathogens exhibiting systemic symptoms being gram-positive cocci. The most prevalent bacteria in this study was *S. aureus*, documented by earlier researchers [9]. This finding is also closely associated with specific indigenous research conducted in the country's southern region, where *S. aureus *was identified as the predominant microbe responsible for generating infections [10]. *P. aeruginosa* is additionally recognized as a pathogenic agent accountable for inducing significant tissue impairments in individuals with diabetes. The researcher demonstrated in a series of 86 samples that *S. aureus* was the predominant pathogen isolated from individuals with diabetes [11]. Additional microbes identified in the study were *P. aeruginosa*, *Proteus mirabilis*, and gram-negative anaerobic microorganisms [12]. The analysis revealed that *S. aureus* was the predominant isolate, followed by *E. coli* and *P. aeruginosa*.

Gram-positive bacteria are frequently the predominant microorganisms identified in various research studies. To effectively manage infections caused by these bacteria, intravenous administration of cefoperazone/sulbactam (SCF) or ceftriaxone was employed as a treatment approach. The accomplishment rate can reach approximately 92%, contingent upon effective care or advancements in the clinical condition. However, numerous other microorganisms were isolated, and the interchange of antibacterial medications occurred based on microbiological findings and sensitivity outcomes. Several antimicrobial medicines were administered, including piperacillin/tazobactam (TZP), clindamycin, vancomycin, and ciprofloxacin.

The study revealed a higher prevalence of diabetes wound affliction among males than among females, consistent with a previous investigation conducted in Karachi, which identified male gender as a contributing factor to diabetic wound infection [13]. Males exhibit a higher susceptibility to injury due to their occupational engagement in outside environments, which exposes them to a broader range of potential hazards. Conversely, females tend to have more limited exposure and comparatively less access to medical treatment. This paper investigates the clinical and microbiological aspects of diabetic wound infections among hospitalized patients in a specific local community. The study focuses on identifying and characterizing common bacteria involved in these infections, with a particular emphasis on their molecular properties. A previous investigation conducted in Pakistan mainly focused on the clinical outcomes of diabetic wound infections [14-16], with most microbiological data derived from various global sources. In the current research investigation, it has been observed that diabetic patients who did not receive antibacterial treatment exhibited the presence of gram-positive and gram-negative species, which were associated with infections of varying severity. In microbiology, it is well observed that diabetic wounds that have been infected tend to exhibit a polymicrobial nature [17]. The wounds of diabetic individuals show variations in the level of infection. Superficial diabetic foot infections typically arise as a result of aerobic gram-positive cocci. In addition, it is worth noting that diabetic wounds often include several microorganisms, including *P. aeruginosa*, Enterobacteriaceae, Enterococci, and anaerobes, frequently observed in such cases [18].

The average age range of individuals at their presentation was between 52 and 74 years, with the age group most significantly impacted being between 41 and 60. Diabetes is prevalent among individuals within commonly observed age categories. Additionally, this age group encompasses those employed and responsible for managing traumatic experiences. As individuals age, they usually have dietary and nutritional inadequacies and a decline in immune function.

The present investigation identified Enterococci, group B Streptococci, *S. aureus*, anaerobic bacteria, and enteric gram-negative bacteria as the microorganisms isolated from cutaneous wounds. The Staphylococcal species accounted for 35.2% of the isolates obtained from wounds of diabetes individuals. The findings of our study are consistent with the results and conclusions reported by researchers (78% and 76%) concerning *S. aureus* [19]. Nevertheless, our investigation needs to demonstrate more robust statistics. As indicated by the literature, the diversity in pathogenic microorganisms may account for the observed differences in ulcer chronicity, degree, and host defense variables.

The predominant microorganisms identified in the study were *S. aureus*, *E. coli*, and *Klebsiella*. A research study conducted in India and subsequently published in the American Diabetic Association in 2006 revealed that *S. aureus* was the most prevalent bacterium in diabetic wound infections, followed by *Proteus*. Additionally, *E. coli* was also detected in these infections [20]. The findings exhibited a resemblance to a prior investigation conducted within the population of the Netherlands [21]. A study conducted in Peshawar a few years ago examined a sample of 114 patients and found that *S. aureus* (46%) was the most prevalent bacterium in diabetic wound infections [22]. A study conducted in China revealed that *Proteus* was the predominant pathogen observed in infected diabetic lesions, followed by *E. coli* [22]. A study conducted in India in 2011 showed that *E. coli* was the most prevalent organism, followed by *S. aureus* [23]. Therefore, *S. aureus* has exhibited the highest prevalence in diabetic wounds during the previous decade. The results of the gram-staining procedure revealed a higher prevalence of gram-negative bacteria compared to gram-positive bacteria. These findings are supported by investigations conducted in India in 2006 [24] and 2011 [25].

In the present investigation, *E. coli* was shown to be the second most commonly isolated organism, accounting for 22.40% of the samples. The pathogenic microorganisms identified in this study included aerobic gram-positive cocci and gram-negative bacilli, such as *E. coli*, *Proteus*, and *Klebsiella* spp. Additionally, it was shown within our sample that there was a high prevalence of both gram-positive and gram-negative infections. In a previous study, researchers exclusively demonstrated the prevalence of gram-positive infections within their respective geographical areas. Comparable findings were documented in research done among the inhabitants of Southern India [26]. Nevertheless, the present investigation revealed a significantly lower abundance of anaerobes than prior reports. Several potential factors could account for the observed outcomes, including delays in transporting samples to the microbiological laboratory and using an incorrect sampling procedure. A higher prevalence of *E. coli* infection has been seen in diabetic wounds. One potential explanation could be the previous administration of antibiotic medications. The correlation between the prior administration of antibacterial medicines to patients and the increased prevalence of drug-resistant strains of *S. aureus* could be a contributing factor. In this investigation, *E. coli* emerged as the second most commonly identified infection in diabetic wounds. The study conducted in India revealed that *E. coli* and *Klebsiella* were the most frequently identified isolates [27].

The antibiotic sensitivity testing revealed that vancomycin had the highest activity level against *S. aureus* and gram-negative aerobes. The use of vancomycin in patients with diabetic nephropathy, a kind of renal illness, may result in detrimental effects due to its exclusive renal clearance. Hence, it is imperative to regulate the dosage appropriately. To make this determination, other alternative antibacterial medications can be considered, such as co-amoxiclav, gentamicin, third-generation cephalosporins, clindamycin, other aminoglycosides, and quinolones. These medications demonstrate varying degrees of vulnerability and resistance to different bacteria that have been found. Sulfamethoxazole/trimethoprim (SXT) had the highest resistance level among antibiotics used in treating diabetic wound infections, followed by cefuroxime and ceftriaxone. The increasing resistance observed can be attributed to the widespread utilization of cephalosporin and sulfamethoxazole/trimethoprim (SXT), more generally referred to as cotrimoxazole, throughout recent decades. This highlights the significance of implementing regulations and surveillance measures for the appropriate utilization of antibiotics based on specific medical situations. Such practices can effectively mitigate the excessive administration of antibiotics, thereby mitigating the development of drug resistance. The efficacy of third-generation cephalosporin against *S. aureus* is limited, with around 23% of strains demonstrating resistance, 48% exhibiting sensitivity, and 29% displaying intermediate resistance. The efficacy of aminoglycosides against *E. coli*, *Pseudomonas*, and, to a certain extent, *S. aureus* has been remarkably noteworthy in terms of sensitivity. However, it is essential to note that aminoglycosides have the potential to cause nephrotoxicity, particularly in those with diabetes who have diabetic nephropathy. Quinolones are not recommended as monotherapy due to their inadequate efficacy against *S. aureus*, Streptococci, and *Klebsiella*. Clinical practitioners must possess awareness regarding the prevalent pathogenic microorganisms found in diabetic wound infections, as well as their respective patterns of antibacterial medication sensitivity. This knowledge is crucial to administer appropriate antibacterial therapy effectively. Therefore, within the scope of this study, it is evident that there is a lack of a singular antibacterial medication capable of effectively targeting all germs. Consequently, a combination of antibiotics must be employed, considering the issue of multidrug resistance (MDR). The emergence of resistant strains poses a multifaceted challenge despite the susceptibility of the microorganism to a specific antibiotic. This is due to the hindered attainment of therapeutic levels of the drug at the infection site, primarily caused by virulence factors such as hemolysins, collagenases, proteases, and short-chain fatty acids. Consequently, this phenomenon gives rise to inflammation and hinders the process of wound healing. This phenomenon exacerbates the persistence of the infection. According to the study, it has been hypothesized that the formation of biofilms in diabetic wounds can hinder the effective penetration of antimicrobial drugs into the diseased region [28].

The researchers have reported that the recognized risk factors for infected diabetic wounds include the duration of diabetes and inadequate control [29,30]. Most patients diagnosed with diabetes in our study had suboptimal control of their condition. Numerous other investigations have corroborated these findings within the context of developing nations. Linezolid (LZD) exhibits efficacy in treating infections caused by gram-positive microorganisms, encompassing strains resistant to methicillin, cephalosporin, and vancomycin [30]. However, its effectiveness against gram-negative organisms is minimal. Nevertheless, linezolid is commonly used to manage recognized microorganisms that have developed resistance to antibacterial drugs due to its relatively high cost. The issue of antibiotic resistance is a significant matter of concern in the field of public health, particularly in developing nations. In some regions, resistance to many medicines has emerged, rendering the existing arsenal of antibiotics useless against various illnesses.

Limitations

However, this study does have a few limitations. The primary limitation of employing a cross-sectional study design is its inherent inability to show causal correlations between diabetic state and wound infections, as it alone captures data at a singular moment in time. Moreover, the reliability of molecular characterization and antibiotic susceptibility testing is contingent upon the quality of laboratory techniques and equipment, which might vary and influence the accuracy of the results. The study's limitations may include omitting certain confounding variables, such as patients' general health conditions and comorbidities, potentially impacting susceptibility to wound infections. Finally, it is essential to note that the study's ability to depict the fluctuating patterns of bacterial resistance over time may be limited. This is because the susceptibility of bacteria to antibiotics might change due to the emergence of new strains and alterations in the usage of antibiotics. Consequently, the study's applicability to future treatment techniques may be constrained.

## Conclusions

The growing problem of antibiotic resistance is a significant matter of public health, particularly in developing nations. In some regions, resistance to many medicines has emerged, rendering the existing arsenal of antibiotics useless against various illnesses. This scenario is a cause for great concern. This work represents a significant advancement in understanding multidrug-resistant (MDR) strains in diabetic patients, offering an updated assessment of the current situation. The findings have important implications for physicians, as they can utilize this information to develop effective methods and guidelines for managing and treating MDR strains in diabetic patients.
